# Automated Cardioailment Identification and Prevention by Hybrid Machine Learning Models

**DOI:** 10.1155/2022/9797844

**Published:** 2022-02-15

**Authors:** K. S. Archana, B. Sivakumar, Ramya Kuppusamy, Yuvaraja Teekaraman, Arun Radhakrishnan

**Affiliations:** ^1^Department of Computer Science and Engineering, Vels Institute of Science, Technology & Advanced Studies (VISTAS), Chennai, India; ^2^Department of Computing Technologies, School of Computing, SRM Institute of Science and Technology, Kattankulathur, Chennai, India; ^3^Department of Electrical and Electronics Engineering, Sri Sairam College of Engineering, City, 562 106, Bangalore, India; ^4^Department of Electronic and Electrical Engineering, The University of Sheffield, Sheffield, S1 3JD, UK; ^5^Faculty of Electrical & Computer Engineering, Jimma Institute of Technology, Jimma University, Ethiopia

## Abstract

Accurate prediction of cardiovascular disease is necessary and considered to be a difficult attempt to treat a patient effectively before a heart attack occurs. According to recent studies, heart disease is said to be one of the leading origins of death worldwide. Early identification of CHD can assist to reduce death rates. When it comes to prediction using traditional methodologies, the difficulty arises in the intricacy of the data and relationships. This research is aimed at applying recent machine learning technology to identify heart disease from past medical data to uncover correlations in data that can greatly improve the accuracy of prediction rates using various machine learning models. Models have been implemented using naive Bayes, random forest algorithms, and the combinations of two models such as naive Bayes and random forest methods. These methods offer numerous attributes associated with heart disease. This proposed system foresees the chance of rising heart disease. The proposed system uses 14 parameters such as age, sex, quick blood sugar, chest discomfort, and other medical parameters which are used in the proposed system. Our proposed systems find the probability of developing heart disease in percentages as well as the accuracy level (accuracy of 93%). Finally, this proposed method will support the doctors to analyze the heart patients competently.

## 1. Introduction

The heart is the only organ that pumps blood to all of the body's tissues via the arteries, veins, and capillaries in order to provide oxygen and nutrition. Vital organs such as the brain and kidney suffer if the heart's pumping motion becomes ineffective, and if the heart stops working entirely, death happens within minutes. Heart disease has been around for a long time, and it has been the most complex and life-threatening human diseases on the planet. Life is beautiful in and out itself. The efficient operation of the heart is fully reliant on it. The following are some of the signs and symptoms of cardiac disease, namely, breathing trouble, physical weakness, left hand paining, and exhaustion are all indicators of heart illness, as are other signals such as high jugular vein pressure and peripheral edema produced by functional cardiac or no cardiac problems. The early inquiry procedures are used to detect the heart disease. Heart problem prevention and therapy are extremely difficult especially in rural areas, due to the scarcity of investigative equipment and specialists, as well as other factors that impede good heart disease prediction and treatment [1].

Nowadays, the artificial intelligence and machine learning are widely acknowledged to show important role in the medical field for diagnosing the disease and classify or forecast the outcomes, it utilizes a variety of machine learning and deep learning models. Machine learning algorithms can quickly adopt thorough genetic data analysis. Medical records may be changed and studied more severely for well estimation, and improved models can be identified for good prediction. Various researchers have reported on the prediction of heart problems using a different algorithm [2].

The common drawback in machine learning is high dimensionality of data which contain large amounts of data and sometimes cannot be seen even in 3D, which is known as the curse of dimensionality. As a result, the overfitting occurs due to more operations done with data analysis and due to this reason, it needed a lot of memory. In addition to reducing redundancy in the dataset, the weighting features can also help reduce the processing time of the execution. The dataset can be reduced in dimensionality using a variety of feature analysis strategies. Hence, the heart disease prediction systems based on machine learning will be precise and reduce risks. This suggested that the proposed algorithm makes a contribution by developing a hybrid machine learning method in medical intelligent decision supporting system for heart disease detection [3].

For this research works, the major contributions are listed below:

- To identify the heart disease, the process involved highly on several key steps such as preprocessing, feature analysis, and finally classification
- A good automated hybrid proposed algorithm model was built to analyze the cardiovascular disease
- This automatic proposed algorithm suggests which features are suitable for designing a good intelligent system for identifying heart disease and healthy people
- Finally, to evaluate the performance, various machine learning models were compared with the proposed algorithm with various similarity metrics to ensure the metrics were improved or not
- This proposed method reduces the human error and achieved very good diagnosis

The remaining sections of the paper are divided into four groups. The introduction is in Section 1, the various related works are in Section 2, Section 3 presents the materials and methods, the result analysis is in Section 4, and the conclusion and future scope are in Section 5.

## 2. Related Work

Several studies have been conducted, and several machine learning models have been used to categories and predict the changes in the heart. Using a machine learning-based technique, various research investigations have reported on the detection of cardiac disease. The classification of performance related to multiple machine learning algorithms on a heart disease dataset was described in a literature study.

Numerous procedures are currently used in heart disease for detection by applying computer vision. The heart disease detection by using and extracting relevant feature with standard dataset used by authors in [1, 4] has been described; the performance of various standard algorithms on the Cleveland heart disease dataset was described. The researchers used the Cleveland heart disease dataset by the University of California Irvine repository. This dataset is used in various researchers which has been utilized to investigate various classification challenges linked to cardiac illnesses using various machine learning classification techniques. The Cleveland dataset was utilized in conjunction with global evolutionary techniques to obtain high prediction accuracy. The characteristics in this study were chosen using feature selection methods. As a result, the approached classification of the performance depends on certain features [5].

The authors in [6] have developed an algorithm for heart disease classification using fusion techniques which combines a fuzzy neural network with an artificial neural network using neural network. The proposed classification system attains an accuracy of 87.4 percent in categorization [7]. SVM approaches for recognizing people with diabetes and then forecasting heart disease had a 94.60% accuracy rate, and the variables employed were common such as blood sugar level, patient's age, and blood pressure data. Dun et al. [8] used a variety of new algorithms and deep learning techniques to diagnose heart illness with hyperparameter tuning to progress the accuracy of the results. The accuracy of neural networks was 78.3 percent, and the other models included logistic regression, SVM, and ensemble approaches like random forest, among others.

According to studies, compared to women's, approximately the males have a heart problem during their lifetime. The higher risk maintained even after correcting for established heart disease risk factors such blood pressure and diabetes. The four important datasets, namely, Cleveland, Switzerland, Hungary, and Long Beach V, are investigated from 1998 by various researchers with important characteristics for heart disease prediction [9].

## 3. Materials and Methods

### 3.1. Dataset

The dataset used in this investigation was the common health dataset, which was created in 1988 in Cleveland. It includes a genuine dataset of 300 data samples with a total of 14 important features (13 predictors, 1 target) such as blood pressure, type of chest discomfort and ECG result as shown in Figure 1. Last but not least, the hybrid algorithm is used to model heart disease and determine the cause of the disease.

### 3.2. Data Preprocessing

Data preprocessing technique is required for the efficient data representation using machine learning, which must be trained and tested thoroughly. For successful use in the classifiers, the preprocessing approaches which follow are missing value removal, standard scalar, and Minmax Scalar. In real life, there are a lot of missing and noisy data to eliminate such errors and produce confident forecasts; the data is preprocessed. Figure 1 shows the successive chart of our proposed model. The standard scalar assures that each feature has the same mean and variance which results in the same coefficient for all features. Minmax Scalar on the other hand adjusts the data so that all features lie in between 0 and 1. The dataset's lost value feature row is simply removed. In this study, all of these data preparation approaches were applied.  Figure 2 shows the complete architecture for identifying heart problem.

### 3.3. Feature Selection

Feature selection is one of the vital roles to select the important feature from the input variable to create a predictive model [9]. From these selected features, the irrelevant features might damage a machine learning classifier for the model performance and this machine learning process necessitates crucial feature selection as shown in Table 1. Relief is a feature selection method that sets weights to all of the dataset's characteristics which allows them to be adjusted over time. The importance of the critical features to target is high, while the importance of the other features is low [10]. For determining feature weights, relief follows the same ideas as K-NN.  Figure 3 shows the selected feature analyzing graph to identify the final heart problem.

### 3.4. Machine Learning Techniques

#### 3.4.1. Naive Bayes Classifier

The naive Bayes classifier is a simple and an effective classification method which is used for creating machine learning models quickly, which can generate accurate predictions. It works by predicting the probability of an object based on its characteristics. It is based on the strong (naive) attribute independence assumption [1]. The Bayes theorem is a mathematical idea that can be used for calculating probabilities as shown in equation (1). There is no relationship or correlation between the predictors. Each of the characteristics contributes to the possibility of maximizing it on its own. It works with the naive Bayes model, but not Bayesian approaches.

(1) $$\begin{array}{c} P\left(\frac{X}{Y}\;\right)=\frac{P\left(Y/X\;\right)\;X\;P\left(X\right)}{P\left(Y\right)}. \end{array}$$

There are four probability expressions in the probability hierarchy: *P*(*X*/*Y*), *P*(*X*), and *P*(*Y*). *P*(*X*) designates the class prior probability, *P*(*Y*) represents the predictor prior probability, and *P*(*Y*) refers to likelihood. In terms of data categorization algorithms, the naive Bayes algorithm is a simple, easy-to-use, nonlinear, and complex approach. However, there is a loss of accuracy because it is based on assumptions and class conditional independence. The dataset's 14 attributes were used to achieve an accuracy of 83.49%.

#### 3.4.2. Random Forest Classifier

A strategy for supervised classification is the random forest algorithm. In this process, several trees are used to form a forest. The random forest emits a class expectation from each tree, and the class with the most votes becomes the model's forecast. A random forest classifier's accuracy improves as the number of trees increases. The following are the three most prevalent methodologies:

- Input choice in random forest
- Random blend forest
- Combination of input choice in random forest and random blend forest

It may be used for classification as well as regression, but it excels in classification and overcomes missing variables [11]. The results are unexplained, aside from being slow to anticipate because of the large datasets and number of trees required. The dataset's 14 attributes were used to achieve an accuracy of 89.20 percent.

#### 3.4.3. Modified Naive Bayes and Random Forest Classifier

The confusion matrix is a performance evaluator for machine learning classification models. The confusion matrix was used to assess the performance of all of the produced models. The confusion matrix shows how many times our models properly predict and how many times they mistakenly guess. True positives and true negatives were assigned to successfully anticipated values, whereas false positives and false negatives were assigned to incorrectly predicted values. The model's performance was evaluated using accuracy, precision, and recall after all of the predicted values were organized in the matrix.

#### 3.4.4. Evaluation Matrices

The confusion matrix is a performance evaluator for machine learning classification models. This calculation assesses the correct performance and shows the performance of the different models. This confusion matrix shows how many times our models properly predict and how many times they mistakenly guess [3]. Here, the true positives and true negatives were assigned to successfully anticipated values, whereas the false positives and false negatives were assigned to incorrectly predicted values as shown in Table 2. Finally, the model's performance was evaluated using accuracy, precision, and recall after all of the predicted values were organized in the matrix [12].

## 4. Results and Discussion

In this section, the final results of different models are discussed below with graphical representation.

### 4.1. Naive Bayes Classifier

Figure 4 shows the predicted result of the confusion matrix of the naive Bayes classifier. The result shows the corrected prediction and the wrong predictions. It has a training accuracy of 83%, test specificity of 84%, and test sensitivity of 86%, respectively.

### 4.2. Random Forest Classifier

Figure 5 shows the matrix calculation and the performance metrics of the existing method of the random forest classifier. The graph depicts the accuracy rate using the ROC curve of prediction of heart disease problem. It has a training accuracy of 89%, test specificity of 85%, and test sensitivity of 84%, respectively.

### 4.3. Modified Naive Bayes and Random Forests

This paper presents a new proposed method of modified naive Bayes and random forest classifier algorithm. It is an extension of the naive Bayes and random forest classifier model. Both these classifiers are used to construct the new classifier algorithm. This classifier gathers all standing instance and classifies new occurrences of similarity based on new correlations through new distance as shown in equation (2). This novelty of our modified naive Bayes and random forest classifier model showed the best results with an accuracy of 92% as shown in Figure 6. This hybrid model can diagnose the heart problem to help the doctors to secure the patients from death.

(2) $$\begin{array}{c} \text{Modified na}\ddot{\text{i}}\text{ve Bayes with random forest classifer}=\sum \sum {\text{dist}}_{\text{corr}\left(\text{a},\text{class}\left(\text{a},\text{b}\right)\right)}. \end{array}$$

The proposed new algorithm is described in Algorithm 1.

### 4.4. Model Comparison Results against Other Existing Methods

Table 3 represents the results of the proposed method of combined naive Bayes and random forest algorithm. This simulation performed in three important performance metrics to identify heart problem. In this simulation, the results show an algorithm to produce better accuracy results compared with existing algorithms of naïve Bayes and random forest classifiers. It has a training accuracy of 92%, test specificity of 85%, and test sensitivity 84%, respectively, as shown in Figure 7.

## 5. Challenges and Future Work

- According to the WHO, the leading death rates globally increased due to the high impact of heart failure in this COVID situation, estimated at 17.9 million in each year, because of high-risk factors such as stress, unhealthy diet, diabetes, blood pressure, and smoking. In many circumstances, preserving a patient's life hinges on the time between seeing a doctor and obtaining the necessary hospitalization, so providing physicians with constant updates on their patients' health status will significantly reduce the number of deaths
- This present work has provided the automatic diagnosis of heart disease prediction and keeps the updated medical status. In the future, the other disorder such as blood pressure, diabetics, and the pulse rate can also be considered related to heart failure and the medical records can also updated using IoT

## 6. Conclusion

The *N* number of patients affected heart problems day by day. So, there is a requirement for a technology that can automatically detect cardiac failure from the symptoms. For this purpose, our proposed algorithm involved various methods to identify heart diseases such as preprocessing, feature extraction, and classification. The dataset has been displayed, and the missing values have been filled in. Some extraneous features have been removed from the data as part of the preprocessing process. Standards were developed to make it easier to incorporate the values into machine learning models. The different performance metrics such as accuracy, recall, and a confusion matrix were utilized to ensure the performance of the proposed model. Finally, this proposed method achieved 92% accuracy compared to other existing methods.

## Figures and Tables

**Figure 1:** Correlation matrix of features in complete dataset.

**Figure 2:** Architecture for identifying heart disease.

**Figure 3:** Feature analysis to identify the heart problem.

**Figure 4:** Confusion matrix and ROC graph of the naïve Bayes classifier.

**Figure 5:** Confusion matrix and ROC graph of the random forest classifier.

**Figure 6:** Confusion matrix and ROC graph of the fusion Naïve Bayes and random forest classifier.

**Figure 7:** Comparison graph of all classifiers.

**Algorithm 1:** Hybrid algorithm to identify the heart problem.

**Table 1:** Feature information and details of the heart disease dataset.

S. no	Feature name	Feature code	Details
1	Patient's age	Age	Patients are calculated in years
2	Patient's sex	Sex	0 = female; 1 = male
3	Variations of chest pain	CP	1—typical angina 2—atypical angina 3—nonanginal pain 4—asymptomatic
4	Level of BP	RBP	mmHg admitted at the hospital
5	Cholesterol status	SCL	Shows cholesterol level in mg/dl
6	Blood sugar fasting > 120 mg/dl	FBS	Fasting blood sugar > 120 mg/dl (0—false; 1—true)
7	Resting electrocardiography	RES	0—normal 1—having ST-T 2—hypertrophy
8	Maximum heart rate	MHR	Over heart rate
9	Exercise-induced angina	EIA	1—yes 0—no
10	ST depression	ST	Exercise to rest
11	ST segment	PES	1—upsloping 2—flat 3—downsloping
12	Size of vessels	VCA	(0–3) colored by fluoroscopy
13	Thalassemia	THA	3—normal 6—static defect 7—dynamic defect
14	Target	Class	0—no risk 1—risk low 2—risk medium 3—risk high 4—danger

**Table 2:** Predicting label of confusion matrix.

Positive	Negative
True positive (TP)	False negative (TN)
False positive (FP)	True negative (FN)

**Table 3:** Performance comparison for various models.

Models	Accuracy (%)	Specificity (%)	Sensitivity (%)
Naïve Bayes classifier	85	84	86
Random forest	89	85	85
Proposed method	92	85	84

## Data Availability

The data used to support the findings of this study are available from the corresponding author upon request.

## References

[1] Sharma V., Yadav S., Gupta M. Heart disease prediction using machine learning techniques.

[2] Al-Jumeily D., Iram S., Vialatte F. B., Fergus P., Hussain A. (2015). A novel method of early diagnosis of Alzheimer’s disease based on EEG signals. *Scientific World Journal*.

[3] Haq A. U., Li J. P., Memon M. H., Nazir S., Sun R., Garciá-Magarinõ I. (2018). A hybrid intelligent system framework for the prediction of heart disease using machine learning algorithms. *Mobile Information Systems*.

[4] Samuel O. W., Asogbon G. M., Sangaiah A. K., Fang P., Li G. (2017). An integrated decision support system based on ANN and Fuzzy_AHP for heart failure risk prediction. *Expert Systems with Applications*.

[5] Edmonds B. Using localised’gossip’to structure distributed learning.

[6] Kahramanli H., Allahverdi N. (2008). Design of a hybrid system for the diabetes and heart diseases. *Expert Systems with Applications*.

[7] Parthiban G., Srivatsa K. (2012). Applying machine learning methods in diagnosing heart disease for diabetic patients. *International Journal of Applied Information Systems*.

[8] Dun B., Wang E., Majumder S. (2016). *Heart disease diagnosis on medical data using ensemble learning, Stanford Publisher*.

[9] Bharti R., Khamparia A., Shabaz M., Dhiman G., Pande S., Singh P. (2021). Prediction of heart disease using a combination of machine learning and deep learning. *Computational Intelligence and Neuroscience*.

[10] Sriram S., Chintagunta P. K. (2010). Learning models. *Marketing Research*.

[11] Martin-Isla C., Campello V. M., Izquierdo C. (2020). Image-based cardiac diagnosis with machine learning: a review. *Frontiers in Cardiovascular Medicine*.

[12] Ghosh M., Raihan M. M. S., Raihan M. (2021). A comparative analysis of machine learning algorithms to predict liver disease. *Intelligent Automation and Soft Computing*.

